The article "Association between the Platelet-Derived Growth Factor/Platelet-Derived Growth Factor Receptor System and Risk of Rheumatoid Arthritis: A Systematic Review and Meta-Analysis" was retracted in 2023. Reasons: unreliable results or conclusions; concerns about the data; concerns about the peer review; concerns about the citations.

# Association between the Platelet-Derived Growth Factor/Platelet-Derived Growth Factor Receptor System and Risk of Rheumatoid Arthritis: A Systematic Review and Meta-Analysis

**DOI:** 10.1155/2022/6221673

**Published:** 2022-03-07

**Authors:** Feiyan Li, Shaoping Wu, Hualing Xie, Wanling Wang, Jing Wang, Chanyi Jia, Chao Xie, Xia Zhang

**Affiliations:** ^1^Department of Rheumatology, Chongqing Hospital of Traditional Chinese Medicine, Chongqing 400021, China; ^2^Department of Cardiology, Chongqing Hospital of Traditional Chinese Medicine, Chongqing 400021, China; ^3^Department of Endocrinology, Chongqing Hospital of Traditional Chinese Medicine, Chongqing 400021, China; ^4^Clinical Support Center, Chongqing Hospital of Traditional Chinese Medicine, Chongqing 400021, China

## Abstract

This research examines the association between the platelet-derived growth factor/platelet-derived growth factor receptor (PDGF/PDGFR) system and rheumatoid arthritis (RA) susceptibility through a comprehensive search of the PubMed database to study the expression of the PDGF/PDGFR system in RA. Review Manager software version 5.3 was used for statistical analysis. Six eligible studies published in the English language were included, including 108 rheumatoid arthritis cases and 85 controls with the corresponding 126 and 97 tests, respectively, relating the expression of the PDGF/PDGFR system to the risk of RA. The overall results indicated a significant association between the PDGF/PDGFR system expression and RA (OR = 5.25, 95% CI: 3.00-9.18, *p* < 00001), RA patients in Asian countries (OR = 4.13, 95% CI = 2.04-8.39, *p* < 0.0001) and in Western countries (OR = 9.18, 95% CI = 2.04-8.39, *p* = 0.03), and only PDGF expression in RA patients (OR = 5.28, 95% CI = 2.73-10.21, *p* < 0.00001). Thus, only the PDGFR expression was insignificantly associated with RA susceptibility (OR = 9.25, 95% CI = 0.63-136.30, *p* = 0.11). Hence, the PDGF/PDGFR system most likely contributes to susceptibility to RA.

## 1. Introduction

Rheumatoid arthritis (RA) is a chronic systemic autoimmune disease with unmet treatment needs that disrupts the lining of the synovial joints, resulting in painful joints and damage to other organs, and can lead to progressive disability, early mortality, and socioeconomic burden [1, 2]. The arm and leg joints affected by RA are characterized by synovial inflammation and hyperplasia, destruction of the bones and cartilages, and production of rheumatoid factor and antibody of anticitrullinated protein with clinical manifestations such as pain, swelling, tenderness, and morning stiffness [2, 3]. Other RA-related conditions are systemic disorders of the pulmonary, cardiovascular, nervous, and skeletal systems [2].

The article "Association between the Platelet-Derived Growth Factor/Platelet-Derived Growth Factor Receptor System and Risk of Rheumatoid Arthritis: A Systematic Review and Meta-Analysis" was retracted in 2023. Reasons: unreliable results or conclusions; concerns about the data; concerns about the peer review; concerns about the citations.

RA symptoms and its treatment goals and outcomes vary from person to person. The diagnosis of RA is employed to categorize the diseases into stages as I, II, III, and IV depending on whether the patient's condition is mild, moderate, severe, and at the end stage, respectively [4, 5]. Treatment options of RA comprise biologic modifiers, receptor-targeted therapies in recognition of the role of cytokines in RA, and medicines for B cell depletion in RA patients [6, 7]. However, therapies for RA treatment are inadequate. As a result, RA patients are faced with a terminal illness that is characterized by progressive destruction of their joints, thereby resulting in pain and poor quality of life [8]. Though reliable biomarkers of RA are few, currently, there are many biomolecules such as anticyclic citrullinated protein antibodies, serum rheumatoid factors, and cytokines that are expressed in the serum and synovial tissues at RA patients' joints and are shown in varying degrees as potential biomarkers of RA [6, 9].

There is a continuing effort to identify candidates of biomarkers in RA, and so far, some biomarkers of RA are likely to be appropriate for target therapy. The platelet-derived growth factor/platelet-derived growth factor receptor (PDGF/PDGFR) system comprises 4 growth factors: PDGFA, PDGFB, PDGFC, and PDGFD, with 2 receptors as PDGFRA and PDGFRB [10]. The PDGF/PDGFR system is associated with rheumatic diseases, cancers, retinal diseases, fibrotic diseases, and cardiovascular diseases [11–13]. Notably, the PDGF/PDGFR system is expressed in RA-fibroblast-like synoviocyte cells and RA-synovial membranes. It is also involved in proliferation and migration and cell morphological changes and has been shown to stimulate the production of matrix metalloproteinases-1 and proinflammatory cytokines in these cells [11, 14–16].

Though the cohorts' studies on the expression of the PDGF/PDGFR are low, there are significant studies of the overexpression of the PDGF/PDGFR system in RA without evidence of any marked association between the PDGF/PDGFR system and RA [14, 17–21]. Therefore, a meta-analysis of the PDGF/PDGFR system's association with RA is needed to develop a fit-for-purpose-targeted treatment of RA. Therefore, this review focuses on assessing the PDGF/PDGFR system's association with rheumatoid arthritis.

## 2. Methods

### 2.1. Identification of Eligible Studies and Data Extraction

A comprehensive search of all English-published literature in June 2021 or earlier, in the PubMed database, to select findings on the expression of platelet-derived growth factors and their receptors in tissues of RA patients and nonarthritic subjects was done for inclusion in this study. The search terms were “platelet-derived growth factor” OR “platelet-derived growth factor receptor” OR “PDGF” or “PDGFR” AND “rheumatoid arthritis.” Two reviewers, LF and WS, independently identified fit-for-purpose studies sequentially by scanning titles/abstracts and reading the full text. All uncertainties and differences were resolved by consensus after rechecking data sources and data conformity to inclusion and exclusion of this research by the third reviewer, WW.

The article "Association between the Platelet-Derived Growth Factor/Platelet-Derived Growth Factor Receptor System and Risk of Rheumatoid Arthritis: A Systematic Review and Meta-Analysis" was retracted in 2023. Reasons: unreliable results or conclusions; concerns about the data; concerns about the peer review; concerns about the citations.

### 2.2. Inclusion and Exclusion Criteria

A study was placed for the meta-analysis to determine if it met the following criteria: (i) it is a case-control study that measured the expression of the platelet-derived growth factors and/or their receptors in the tissues of nonarthritic and RA patients and (ii) it contained original and sufficient data to calculate odds ratios (ORs). For exclusion criteria of studies, the following was used: (i) studies in which the number of study participants could not be ascertained, (ii) relevant studies in which there is no sufficient data to estimate the number of patient samples that showed significant expression of PDGF and/or PDGFR, (iii) studies using only cell lines and/or animal models or research that is unrelated to the objectives of this study, and (iv) review, expert opinions, editorials, conference abstracts, letters, and case reports involving 1 patient.

### 2.3. Data Extraction

The first and second reviewers detailed the expression of PDGF and/or PDGFR in the tissues of RA patients and the control, which are nonarthritic subjects from eligible publications using a standard and relevant data extraction form and presented in an orderly manner to facilitate easy comparison and analysis of the extracted data. The following information was collected from the eligible research for the meta-analysis: the surname of the first author, year of publication, country of location of the study subjects, the number RA and control subjects, the cohort of the study, estimation of the number of study RA, and the control study subjects that have shown to express PDGF and/or PDGFR from graphs and tables. All the data were recorded in an Excel spreadsheet for analysis.

### 2.4. Statistical Analysis

Meta-analysis was done, employing the Review Manager version 5.3 to determine the significance of the association between susceptibility of RA and the expression of the PDGF/PDGFR system in the tissues of RA patients. This was analyzed using the estimated OR of all the eligible studies at a 95% confidence interval (CI). In addition, the pooled effect sizes were obtained from forest plots of the OR of individual studies at 95% CI to evaluate the association between expression and no expression of the PDGF/PDGFR system among combined dichotomous sets of RA and nonarthritic subjects. The forest plots gave the overall effect of growth factors (PDGF) and their receptors (PDGFR) on RA, the effect of only PDGF and only PDGFR on RA, and the effect size of study subjects in Western and Asian studies countries has been analyzed. An OR less than 1, equal to 1, and greater than 1 showed minor association, no association, and a more significant association between the expression of the PDGF/PDGFR system in the tissues of RA patients over nonarthritic subjects.

The article "Association between the Platelet-Derived Growth Factor/Platelet-Derived Growth Factor Receptor System and Risk of Rheumatoid Arthritis: A Systematic Review and Meta-Analysis" was retracted in 2023. Reasons: unreliable results or conclusions; concerns about the data; concerns about the peer review; concerns about the citations.

To estimate OR, a fixed-effect Mantel-Haenszel model was employed in the beginning. Where the *I*^2^ statistic was greater than 50% or the *p* value was less than 0.10, it was interpreted as significant heterogeneity across studies; therefore, further analysis was done, using the random-effect model to estimate the pooled effect. Additionally, funnel plots were used to investigate potential biases that might stem from the publications.

## 3. Results

### 3.1. Publications Search

Figure 1 details an outline of the data search and the selection of studies in this research. An examination of the PubMed database showed 200 studies, of which 179 were excluded based on the inclusion criteria after scanning the titles and abstracts of 200 articles. A full-text perusal of the remaining 39 studies led to the selection of 6 studies for the meta-analysis. The remaining 15 studies were excluded due to insufficient data to allow data extraction for the analysis. For the 6 studies included in the meta-analysis, 1 study of patients in a Western country had 4 datasets on the PDGFA, PDGFB, PDGFC, and PDGFD [17]. Thus, the 6 studies had 9 datasets drawn from 6 countries, comprising 3 Western countries and 3 Asian countries. The 4 datasets of one of the 6 studies were treated separately by placing “pdgfA,” “pdgfB,” “pdgfC,” and “pdgfD” in parentheses against the surname of the first author of this study.

The association between susceptibility to RA and the PDGF/PDGR system expression was meta-analyzed using the 6 studies with 9 datasets, as shown in Table 1 and Figure 2. Additionally, subgroup meta-analysis of susceptibility to RA and only PDGFR and only PDGF expression from 3 studies with 3 datasets and 3 studies with 6 datasets, respectively, were undertaken. The 6 studies with 9 datasets had 90 of 126 tests of RA and 27 of 97 tests of nonarthritic subjects had records of PDGF/PDGFR system expression. For only PDGFR and only PDGF, 32 of 43 tests of RA and 6 of 21 tests of nonarthritic subjects were analyzed for only PDGFR. In contrast, 58 of 83 tests of RA and 21 of 76 tests for nonarthritic subjects had records of expression of only PDGF. Furthermore, comparing the susceptibility to RA due to PDGF/PDGFR system expression among patients in Western countries and Asian countries was meta-analyzed using 3 studies with 6 datasets and 3 other studies with 3 datasets, respectively. For the expression of the PDGF/PDGFR system in Asian and Western countries, 51 of 77 tests of RA and 21 of 65 nonarthritic subjects were recorded in Asian countries, while Western countries had 39 of 49 tests of RA patients and 6 of 32 tests of nonarthritic subjects.

The article "Association between the Platelet-Derived Growth Factor/Platelet-Derived Growth Factor Receptor System and Risk of Rheumatoid Arthritis: A Systematic Review and Meta-Analysis" was retracted in 2023. Reasons: unreliable results or conclusions; concerns about the data; concerns about the peer review; concerns about the citations.

### 3.2. The Association between PDGF/PDGFR Expression and Susceptibility to RA

An overview of the associations between PDGF/PDGFR system expression and RA is provided in Figures 2 and 3.

Six studies with 9 datasets were included in the meta-analysis to evaluate the association between PDGF/PDGFR system expression and RA subjects in Figure 2. The *I*^2^ and *p* value for heterogeneity were 43% and 0.08, respectively. Among the RA and nonarthritic subjects, the PDGF/PDGFR system expression had 5.25 highly significant greater odds of association in RA patients than the nonarthritic subjects. Thus, the meta-analysis showed a more significant association between PDGF/PDGFR system expression and RA patients in the overall population of the study (OR = 5.25, 95% CI = 3.00-9.18, *p* < 00005).

Figures 3(a) and 3(b) show the meta-analysis of associations of only PDGFR expression and only PDGF expression on the one hand and PDGF/PDGFR system expression in RA patients examined in Asian countries and Western countries on the other hand in Figures 3(c) and 3(d). To evaluate the association between only PDGFR expression and the RA patients, 3 studies with 3 datasets were included in the meta-analysis. The *I*^2^ and *p* value for heterogeneity were 63% and 0.07, respectively. Therefore, further analysis was performed using the random-effect model. As a result, the PDGFR expression in RA patients has 9.25 insignificant greater odds of association than that in nonarthritic subjects, as shown in the meta-analysis (OR = 9.25, 95% CI = 0.63-136.30, *p* = 0.11). In contrast, studies of PDGF expression in RA and nonarthritic subjects revealed the *I*^2^ and the *p* value for heterogeneity to be 42% and 0.13, respectively. Also, there was a significantly high PDGF expression with a 5.28 greater odds of association with RA patients compared with nonarthritic subjects, as shown in Figure 3(b) of the meta-analysis (OR = 5.28, 95% CI = 2.73-10.21, *p* < 0.00001).

For the assessment of the association between PDGF/PDGFR system expression and RA susceptibility of patients in Asian countries, 3 studies with 3 datasets were meta-analyzed. The *I*^2^ and the *p* value for heterogeneity were 0% and 0.65, respectively. The odds of association of the PDGF/PDGFR system expression in RA patients were 4.13, more significant than that in the nonarthritic group in Figure 3(c) of the meta-analysis (OR = 4.13, 95% CI = 2.04-8.39, *p* < 0.0001). In contrast, the association between PDGF/PDGFR system expression and RA subjects in Western countries involved 3 studies with 6 datasets. Records of the *I*^2^ and the *p* value for heterogeneity were 61% and 0.02, respectively.

The article "Association between the Platelet-Derived Growth Factor/Platelet-Derived Growth Factor Receptor System and Risk of Rheumatoid Arthritis: A Systematic Review and Meta-Analysis" was retracted in 2023. Reasons: unreliable results or conclusions; concerns about the data; concerns about the peer review; concerns about the citations.

Further analysis was done using the random-effect model. As a result, the association between PDGF/PDGFR system expression in RA patients located in Western countries has 9.18 odds of significant association than that in the nonarthritic group as shown in Figure 3(d) of the meta-analysis (OR = 9.18, 95% CI = 2.04-8.39, *p* = 0.03). Thus, the analysis has shown that the odds of association of the PDGF/PDGFR system expression in RA patients are higher among Western countries than in Asian countries.

### 3.3. Publication Bias

The analyses of PDGF/PDGFR system expression in RA patients and the nonarthritic group demonstrated that all the studies included in the meta-analysis showed significantly higher odds of associations among RA patients than the nonarthritic group in the overall population of the study subjects. Additionally, the funnel plot analysis for the 6 studies with 9 datasets was included in the meta-analysis, as shown in Figure 4. The symmetrical shape of the funnel plot does not indicate any publication bias though most of the sample population of eligible studies for the meta-analysis was small.

## 4. Discussion

Several studies evaluating the role of cytokine protein array profile associated with RA have been done with varied outcomes of these cytokines, including the PDGF/PDGFR system that calls for developing and integrating cytokine-targeted treatments for RA disease in the future [6, 22–24]. Invariably, the meta-analyses of cytokines implicated in the development and progression of RA disease are needed to develop a fit-for-purpose-targeted treatment for RA disease.

The PDGF/PDGFR system has shown its immense role in the development and progression of RA disease as follows: several pieces of research on the PDGF/PDGFR system in tissues of RA patients and in vitro and in vivo studies have demonstrated the system's significant role in the occurrence, development, and progression of RA. The PDGF is known to play a crucial role in proliferation and migration, cause an increase in mRNA and protein expressions of proinflammatory cytokines such as interleukin-1b and interleukin-8 by synergizing with the tumor necrosis factor in the RA-fibroblast-like synoviocytes (FLS), increased the amounts of FLS in the G2/M cell cycle phase, promote morphological changes of the FLS cells to a dendritic shape, and cause a significant increase in cathepsin B secretion that can degrade some collagen types and proteoglycans in acidic physiological conditions [14, 16, 20, 21, 25–32]. Furthermore, the mechanism of PDGF's role in proliferation and migration results from synergistic action between PDGF and interleukin-1 in indomethacin [26]. There are also reports of association of the PDGFR with chronic synovial inflammation and involvement in the development of the destructive phenotype of synovial cells in RA [17, 19].

The article "Association between the Platelet-Derived Growth Factor/Platelet-Derived Growth Factor Receptor System and Risk of Rheumatoid Arthritis: A Systematic Review and Meta-Analysis" was retracted in 2023. Reasons: unreliable results or conclusions; concerns about the data; concerns about the peer review; concerns about the citations.

These reports call for a meta-analysis to ascertain the level of significance of the PDGF/PDGFR system expression with RA susceptibility. The data from published pieces of research were combined to evaluate the overall association of PDGF/PDGFR system expression in RA patients and subgroup analysis of the system's association with RA based on the in-country location of the patients, and the association of only the PDGFs and only PDGFR with RA was evaluated. We discovered significant associations of the PDGF/PDGFR system expression with RA patients across the entire population of all the study subjects and with RA patients in Asian countries and Western countries and marked the association between only PDGF expression with RA patients than with control subjects. Thus, only PDGFR expression in the study subject was insignificantly associated with RA susceptibility. It is worth noting that although there was more tests of the PDGF/PDGFR system expression in the study subjects of Asian countries with 142 tests than in the study subjects of Western countries with 81 tests, the association of PDGF/PDGFR system expression was more associated with RA patients in Western countries than in Asian countries.

In addition, the testing for only PDGF and only PDGFR recorded 64 tests and 159 tests, respectively. Hence, the vast difference in the numbers might have accounted for the insignificance of the association between only PDGFR with RA susceptibility. However, overall, the population of the study subjects was small. Therefore, we recommend that more large sample sizes for the study of PDGF/PDGFR system expression in RA patients should be done in the future, with attention to details on the country of origin of RA patients to allow concrete evaluation of ethnic-origin RA patients PDGF/PDGFR system expression association with RA susceptibility.

This meta-analysis is the first of its kind to ascertain the PDGF/PDGFR system expression with RA susceptibility. Considering that the PDGF/PDGFR system expression in human adults is associated with diseases and also has a significant association with RA, then targeting this PDGF/PDGFR has great potential in the design of combination therapies for RA [10].

The article "Association between the Platelet-Derived Growth Factor/Platelet-Derived Growth Factor Receptor System and Risk of Rheumatoid Arthritis: A Systematic Review and Meta-Analysis" was retracted in 2023. Reasons: unreliable results or conclusions; concerns about the data; concerns about the peer review; concerns about the citations.

## 5. Conclusion

The overall results indicated a significant association between the PDGF/PDGFR system expression and RA, with a higher association among RA patients in Western countries than in Asian countries. Additionally, only PDGF expression in RA patients showed a significant association, while only PDGFR expression in RA patients was not significantly associated with RA susceptibility. In conclusion, the findings in this meta-analysis suggest that the PDGF/PDGFR system expression is significantly associated with RA susceptibility, especially the PDGFs, and more significantly associated with RA patients in Western countries. The limitation of this study is few cohorts. However, these findings present evidence that calls for large cohort studies in PDGF/PDGFR system expression in RA to pave the way for a comprehensive updated investigation in the future.

## Figures and Tables

**Figure 1:** PRISMA flow diagram of comprehensive literature search and details of selected eligible studies for inclusion in PDGF/PDGFR system expression meta-analysis. The PRISMA Statement. PLoS Med 6(6): e1000097. doi:10.1371/journal.pmed1000097

**Figure 2:** Odd ratios at 95% CI of individual studies and pooled data for the association between PDGF/PDGFR system expression and RA in all studies.

**Figure 3:** Odd ratios at 95% CI of individual studies and pooled data for the association between expression of only PDGFR (a) and only PDGF (b) expression with RA and association of PDGF/PDGFR system expression within subjects of Asian (c) and Western (d) countries.

**Figure 4:** Funnel plot for assessing publication bias in the meta-analysis of the 6 studies for PDGF/PDGFR system expression and susceptibility to the RA disease.

**Table 1:** Characteristics of respective studies included in the meta-analysis.

Author	Year	Country	Rheumatoid arthritis (RA)	Control/nonarthritis (NA)	Cohort	Sample	Detection	Gene	PDGF/PDGFR expression (RA)	PDGF/PDGFR expression (NA)
Rubin	1988	Sweden	15	5	20	STB	IHC	PDGFR	15	0
Watanabe	2002	Japan	3	3	6	STB	RT-PCR	PDGFRA	2	1
Walsh	2010	UK	10	11	21	CSMTMTP	IHC	PDGFB	10	0
Charbonneau (pdgfA)	2016	Canada	6	4	10	STB	IHC	PDGFA	2	2
Charbonneau (pdgfB)	2016	Canada	6	4	10	STB	IHC	PDGFB	4	1
Charbonneau (pdgfC)	2016	Canada	6	4	10	STB	IHC	PDGFC	4	1
Charbonneau (pdgfD)	2016	Canada	6	4	10	STB	IHC	PDGFD	4	2
Matsumura	2019	Japan	25	13	38	STB	IHC	PDGFRA/B	15	5
Wang	2020	China	49	49	98	VWB	ELISA	PDGFB	34	15

VWB: venous whole blood; STB: synovial tissue biopsy; CSMTMTP: coronal section of middle third of medial tibial plateaux; ELISA: enzyme-linked immunosorbent assay; IHC: immunohistochemistry; RT-PCR: real-time polymerase chain reaction.

The article "Association between the Platelet-Derived Growth Factor/Platelet-Derived Growth Factor Receptor System and Risk of Rheumatoid Arthritis: A Systematic Review and Meta-Analysis" was retracted in 2023. Reasons: unreliable results or conclusions; concerns about the data; concerns about the peer review; concerns about the citations.

## Data Availability

No data were used to support this study.

## References

[1] Guo Q., Wang Y., Xu D., Nossent J., Pavlos N. J., Xu J. (2018). Rheumatoid arthritis: pathological mechanisms and modern pharmacologic therapies. *Bone Research*.

[2] McInnes I. B., Schett G. (2011). The pathogenesis of rheumatoid arthritis. *New England Journal of Medicine.*.

[3] Van Holsbeeck M., Van Holsbeeck K., Gevers G. (1988). Staging and follow-up of rheumatoid arthritis of the knee. Comparison of sonography, thermography, and clinical assessment. *Journal of Ultrasound in Medicine*.

[4] Schroecksnadel K., Winkler C., Duftner C., Wirleitner B., Schirmer M., Fuchs D. (2006). Tryptophan degradation increases with stage in patients with rheumatoid arthritis. *Clinical Rheumatology.*.

[5] Lovering C. (2021). Four stages and progression of rheumatoid arthritis.

[6] Feldmann M., Brennan F. M., Maini R. N. (1996). Role of cytokines in rheumatoid arthritis. *Annual Review of Immunology.*.

[7] Goldblatt F., Isenberg D. (2005). New therapies for rheumatoid arthritis. *Clinical & Experimental Immunology.*.

[8] Willkens R. F. (1991). Prognostic staging for therapy of rheumatoid arthritis. *Seminars in Arthritis and Rheumatism*.

[9] Wu T., Sajitharan D., Mohan C. (2010). Biomarkers of rheumatoid arthritis: recent progress. *Expert Opinion on Medical Diagnostics.*.

[10] Reigstad L. J., Varhaug J. E., Lillehaug J. R. (2005). Structural and functional specificities of PDGF-C and PDGF-D, the novel members of the platelet-derived growth factors family. *The FEBS Journal.*.

[11] Kameda H., Suzuki M., Takeuchi T. (2007). Platelet-derived growth factor as a therapeutic target for systemic autoimmune diseases. *Drug Target Insights*.

[12] Manzat Saplacan R. M., Balacescu L., Gherman C. (2017). The role of PDGFs and PDGFRs in colorectal cancer. *Mediators of Inflammation*.

[13] Andrae J., Gallini R., Betsholtz C. (2008). Role of platelet-derived growth factors in physiology and medicine. *Genes & Development*.

[14] Wang B.-H., Lu Y.-H., Wu L.-F. (2020). Evaluation of plasma cytokine protein array profile: the highlighted PDGF-BB in rheumatoid arthritis. *Clinical Rheumatology*.

[15] Pohlers D., Huber R., Ukena B., Kinne R. W. (2006). Expression of platelet-derived growth factors C and D in the synovial membrane of patients with rheumatoid arthritis and osteoarthritis. *Arthritis and Rheumatism*.

The article "Association between the Platelet-Derived Growth Factor/Platelet-Derived Growth Factor Receptor System and Risk of Rheumatoid Arthritis: A Systematic Review and Meta-Analysis" was retracted in 2023. Reasons: unreliable results or conclusions; concerns about the data; concerns about the peer review; concerns about the citations.

[16] Bergström B., Carlsten H., Ekwall A.-K. H. (2018). Methotrexate inhibits effects of platelet-derived growth factor and interleukin-1*β* on rheumatoid arthritis fibroblast-like synoviocytes. *Arthritis Research & Therapy*.

[17] Charbonneau M., Lavoie R. R., Lauzier A., Harper K., McDonald P. P., Dubois C. M. (2016). Platelet-derived growth factor receptor activation promotes the prodestructive invadosome-forming phenotype of synoviocytes from patients with rheumatoid arthritis. *The Journal of Immunology.*.

[18] Matsumura T., Saito Y., Suzuki T. (2019). Phosphorylated platelet-derived growth factor receptor-positive cells with anti-apoptotic properties accumulate in the synovium of patients with rheumatoid arthritis. *Frontiers in Immunology.*.

[19] Rubin K., Terracio L., Rönnstrand L., Heldin C. H., Klareskog L. (1988). Expression of platelet-derived growth factor receptors is induced on connective tissue cells during chronic synovial inflammation. *Scandinavian Journal of Immunology*.

[20] Walsh D. A., McWilliams D. F., Turley M. J. (2010). Angiogenesis and nerve growth factor at the osteochondral junction in rheumatoid arthritis and osteoarthritis. *Rheumatology*.

[21] Watanabe N., Ando K., Yoshida S. (2002). Gene expression profile analysis of rheumatoid synovial fibroblast cultures revealing the overexpression of genes responsible for tumor-like growth of rheumatoid synovium. *Biochemical and Biophysical Research Communications.*.

[22] McInnes I. B., Schett G. (2007). Cytokines in the pathogenesis of rheumatoid arthritis. *Nature Reviews Immunology.*.

[23] Lubberts E., van den Berg W. B. (2013). *Cytokines in the pathogenesis of rheumatoid arthritis and collagen-induced arthritis*.

[24] Alunno A., Carubbi F., Giacomelli R., Gerli R. (2017). Cytokines in the pathogenesis of rheumatoid arthritis: new players and therapeutic targets. *BMC Rheumatology*.

[25] Cheon H., Sun Y., Yu S. (2004). Platelet-derived growth factor-AA increases IL-1beta and IL-8 expression and activates NF-kappaB in rheumatoid fibroblast-like synoviocytes. *Scandinavian Journal of Immunology*.

[26] Kumkumian G. K., Lafyatis R., Remmers E. F., Case J. P., Kim S., Wilder R. L. (1989). Platelet-derived growth factor and IL-1 interactions in rheumatoid arthritis. Regulation of synoviocyte proliferation, prostaglandin production, and collagenase transcription. *Journal of Immunology, Virus Research and Experimental Chemotherapy*.

[27] Kameda H., Ishigami H., Suzuki M., Abe T., Takeuchi T. (2006). Imatinib mesylate inhibits proliferation of rheumatoid synovial fibroblast-like cells and phosphorylation of gab adapter proteins activated by platelet-derived growth factor. *Clin Exp Immunol*.

The article "Association between the Platelet-Derived Growth Factor/Platelet-Derived Growth Factor Receptor System and Risk of Rheumatoid Arthritis: A Systematic Review and Meta-Analysis" was retracted in 2023. Reasons: unreliable results or conclusions; concerns about the data; concerns about the peer review; concerns about the citations.

[28] Shimozato O., Watanabe N., Goto M., Kobayashi Y. (1996). Cytokine production by SV40-transformed adherent synovial cells from rheumatoid arthritis patients. *Cytokine*.

[29] Migita K., Eguchi K., Aoyagi T. (1996). The effects of the immunosuppressant rapamycin on the growth of rheumatoid arthritis (RA) synovial fibroblast. *Clin Exp Immun*.

[30] Wang H., Fang Y., Wang Y. (2012). Clinical pathways based on integrative medicine in chinese hospitals improve treatment outcomes for patients with acute myocardial infarction: a multicentre, nonrandomized historically controlled trial. *Evidence-Based Complementary and Alternative Medicine*.

[31] Marcinkiewicz J., Gluszko P., Kontny E. (2007). Is Taurolidine a candidate for treatment of rheumatoid arthritis?. *Clinical and Experimental Rheumatology.*.

[32] Lemaire R., Huet G., Zerimech F. (1997). Selective induction of the secretion of cathepsins B and L by cytokines in synovial fibroblast-like cells. *Rheumatology*.

